The article "Effects of a Brain-Computer Interface-Operated Lower Limb Rehabilitation Robot on Motor Function Recovery in Patients with Stroke" was retracted in 2023. Reasons: signs of a paper mill; suspected computer-generated content; unreliable results or conclusions; concerns about the data.

# Effects of a Brain-Computer Interface-Operated Lower Limb Rehabilitation Robot on Motor Function Recovery in Patients with Stroke

**DOI:** 10.1155/2021/4710044

**Published:** 2021-12-20

**Authors:** Chao Li, Jinyu Wei, Xiaoqun Huang, Qiang Duan, Tingting Zhang

**Affiliations:** ^1^Department of Neurology, The People's Hospital of China Three Gorges University.The First People's Hospital of Yichang, Yichang, China; ^2^Department of Ultrasound, Yichang Maternity & Child Healthcare Hospital. Yichang Children's Hospital, Yichang, China; ^3^Department of Rehabilitation Medicine, The People's Hospital of China Three Gorges University.The First People's Hospital of Yichang, Yichang, China; ^4^Department of Radiology, The People's Hospital of China Three Gorges University.The First People's Hospital of Yichang, Yichang, China

## Abstract

**Purpose:**

To observe the effect of a brain-computer interface-operated lower limb rehabilitation robot (BCI-LLRR) on functional recovery from stroke and to explore mechanisms.

**Methods:**

Subacute-phase stroke patients were randomly divided into two groups. In addition to the routine intervention, patients in the treatment group trained on the BCI-LLRR and underwent the lower limb pedal training in the control group, both for the same time (30 min/day). All patients underwent assessment by instruments such as the National Institutes of Health Stroke Scale (NIHSS) and the Fugl–Meyer upper and lower limb motor function and balance tests, at 2 and 4 weeks of treatment and at 3 months after the end of treatment. Patients were also tested before treatment and after 4 weeks by leg motor evoked potential (MEP) and diffusion tensor imaging/tractography (DTI/DTT) of the head.

**Results:**

After 4 weeks, the Fugl–Meyer leg function and NIHSS scores were significantly improved in the treatment group vs. controls (*P* < 0.01). At 3 months, further significant improvement was observed. The MEP amplitude and latency of the treatment group were significantly improved vs. controls. The effect of treatment on fractional anisotropy values was not significant.

**Conclusions:**

The BCI-LLRR promoted leg functional recovery after stroke and improved activities of daily living, possibly by improving cerebral-cortex excitability and white matter connectivity.

## 1. Introduction

The recovery of neuronal function after central nervous system injury is very difficult. How to regenerate defective neurons and restore the conduction function of axons has been a medical problem worldwide. With the development of multidisciplinary techniques such as neuroscience, signal detection, pattern recognition, and external assistive technologies (e.g., lower limb rehabilitation robots and brain-computer interfaces), the progress study of leg motion control and walking function after central nervous system injury has been ascensively made and become a research hotspot in recent years [1].

The article "Effects of a Brain-Computer Interface-Operated Lower Limb Rehabilitation Robot on Motor Function Recovery in Patients with Stroke" was retracted in 2023. Reasons: signs of a paper mill; suspected computer-generated content; unreliable results or conclusions; concerns about the data.

The BCI-LLRR is a new idea for the recovery of limb motor function in patients with stroke [2]. However, many questions concerning this approach remain unanswered. Relevant clinical case reports are rare, effective evaluation and testing standards are not uniform, and the safety and effectiveness of long-term treatment are not clear [3, 4]. In a previous research project, we constructed a brain-based, active-passive, and stimulating lower limb rehabilitation robot operated and clinically observed the functional recovery of patient, users with stroke. Here, we report further on the clinical application of our system in patients with stroke.

## 2. Materials and Methods

### 2.1. General Information

A total of thirty-three patients were enrolled in this study. Seven patients were excluded because of age, duration of disability, or comorbid cognitive impairment. One patient was discontinued due to an adverse reaction. Twenty-five patients were included in the analysis, comprising thirteen patients in the control group and twelve in the treatment group (Figure 1). And there was no significant difference in gender, age, and duration between the two groups (Table 1). All work was conducted with the principles of the Declaration of Helsinki.

### 2.2. Inclusion Criteria

(1) First onset, in line with the criteria for diagnosis and classification of strokes formulated by the Chinese Neuroscience Society and the Chinese Society of Neurosurgery at the Sixth National Cerebrovascular Disease Conference 2004. (2) Diagnosis by computed tomography or MRI of cerebral haemorrhage or cerebral infarct in cortex or a subcortical area confined to one hemisphere. (3) Vital signs stable, consciousness unimpaired, and no aphasia. (4) Included in the study between 2 weeks and 6 months after onset. (5) Aged between 30 and 70 years. (6) Hemiplegic motor dysfunction. (7) Informed consent signed with the patient or family before treatment.

### 2.3. Exclusion Criteria

(1) Unstable condition due to progressive or secondary brain injury; (2) presence of skull defects or metal implants in the skull; (3) history of epilepsy; (4) presence of unilateral neglect; (5) history of eye disease affecting vision; (6) history of cerebral vascular disease, craniocerebral injury, or peripheral neuropathy; (7) history of severe mental or pulmonary dysfunction; (8) limb dysfunction due to other causes, including nerve, muscle, or bone damage; (9) had participated in BCI-operated lower limb rehabilitation<6 months prior to the study.

The article "Effects of a Brain-Computer Interface-Operated Lower Limb Rehabilitation Robot on Motor Function Recovery in Patients with Stroke" was retracted in 2023. Reasons: signs of a paper mill; suspected computer-generated content; unreliable results or conclusions; concerns about the data.

### 2.4. Treatment Method

All patients admitted to the hospital received medication for blood pressure control, lipid-lowering statins, nutrition supporting nerve function, and symptomatic supportive treatment. Blood pressure was stable in all cases. Both groups of patients received routine rehabilitation interventions (including limb compression, intermediate-frequency, pulsed electrical therapy, and partial hemiplegia comprehensive training). The treatment group received supplementary training on the BCI-LLRR once per day for 30 min, while without image, video, and sound hint in the control group. All treatments were operated by trained technicians, providing safety for the experiment, and those works were performed once per day for 4 weeks.

### 2.5. The BCI-LLRR

The verification platform system of the BCI-LLRR is a vital power integration system based on the distributed heterogeneous device interface of COM and the heterogeneous device integration of Ethernet. In the rehabilitation robot, the feedback compensation control technology based on motion information is added, that is, the signal collected by light point motion, body sensor, and pressure sensor is input to a new hybrid controller based on the combination of man-machine coupling impedance control method and the bang-bang control method to realize the motion feedback compensation of the lower limb intelligent training rehabilitation robot.

### 2.6. Clinical Scales for Evaluation of Function

All patients underwent rehabilitation assessment after admission at 2 and 4 weeks of treatment, using the National Institutes of Health Stroke Scale (NIHSS), the Fugl–Meyer scale (upper and lower limb), the Fugl–Meyer balance scale, and the Holden walking function assessment. The NIHSS scale is used to assess the extent of nerve damage in patients with stroke. The Fugl–Meyer scale includes an upper and lower extremity exercise scale for assessing the patient's motor function. The Fugl–Meyer balance scale is divided into scales for sitting and standing balance. The Holden scale assesses walking ability. Lower NIHSS scores are better; in all other instruments, higher scores are better recovery. All of the above evaluations were performed by a therapist blinded to the patient's treatment plan.

### 2.7. Objective Functional and Structural Status Indicators

All patients were examined using the characteristics of the leg motor evoked potential (MEP) with recording by an electromyography system (MEB-9404, Japan Optoelectronics Co., Ltd.) and stimulation by magnetic stimulator (YRD CCY-1, Wuhan Erideide Co., Ltd.). Diffusion tensor imaging/tractography (DTI/DTT; Signa 1.5 T superconducting magnetic resonance imager, GE, Wisconsin, USA) was used to evaluate the condition of the corticospinal tract (CST). We observed the MEP amplitude, the MEP latency, and the CST for changes before and after 4 weeks of treatment. The outer diameter of the stimulation coil was 10.5 cm and the maximum output intensity was 2.5 T. The stimulation point was 5 cm in front of the Cz point of the head, and the stimulation strength was 90% of threshold for contraction of the tibialis anterior muscle. The participant was placed in the supine position and recording electrodes were placed on the skin over the bellies and the tibialis anterior muscles of both legs. The anode was placed distally to the cathode, the distance between the anode and cathode was 2 cm, and the impedance between the electrodes was less than 5 kΩ. The signal was amplified and recorded by the electromyograph. The measurement was repeated multiple times with a potential high enough for reproducibility and the maximum amplitude and minimum peak latency determined. Higher amplitudes and lower latencies are better.

The article "Effects of a Brain-Computer Interface-Operated Lower Limb Rehabilitation Robot on Motor Function Recovery in Patients with Stroke" was retracted in 2023. Reasons: signs of a paper mill; suspected computer-generated content; unreliable results or conclusions; concerns about the data.

All patients underwent DTI/DTT scans with an 8-channel skull coil, including axial-position T1, T2 weighting, FLAIR, and axial-position, sagittal-position, and coronal-position T1WI. The parameters of DTI/DTT were SE-EPI sequence, TR, 8000 ms, TE, 97.7–98.3 ms, layer thickness, 5.0 mm, layer spacing, 0 mm, matrix, 128 × 130, field of view, 24 cm × 24 cm, excitation times, 1, *b*, 0 and 1000 s/mm^2^, and 15 diffusion-sensitive gradient directions. The obtained image was processed by Functool software to obtain the fractional anisotropy (FA) map. The researchers manually mapped the region of interest on the ipsilateral and lesion side to the contralateral side to obtain a denominator for calculating the FA. Higher FAs are better. All the examiners were blind of the patient's group.

### 2.8. Statistical Analysis

The data are expressed as mean ± standard deviation, and the raw data were statistically analysed using SPSS 21.0 software, including paired *t*-test, repeated-measures' analysis of variance and chi-square test. *P* < 0.05 was considered to indicate a significant difference.

## 3. Results

### 3.1. Function Assessments

Both the Fugl–Meyer (lower limb) and NIHSS scores were significantly improved at 2 weeks and 4 weeks (*P* < 0.05) (Figures 2(a) and 2(b)), while the Fugl–Meyer (upper limb), Fugl–Meyer balance, and Holden scores were not significantly improved (*P* > 0.05). Compared with the control group, the Fugl–Meyer (lower limb) scores were significantly improved in the treatment group after 2 weeks (*P* < 0.05) (Figure 2(b)) and 4 weeks (*P* < 0.01). The NIHSS scores were also significantly improved in the treatment group after 4 weeks (*P* < 0.01) (Figures 2(a) and 2(b)). At follow-up, scores on the Fugl–Meyer balance scales (Figure 3(a)) and Holden walking tests (Figure 3(b)) are significantly increased compared with the control group (*P* < 0.05).

The article "Effects of a Brain-Computer Interface-Operated Lower Limb Rehabilitation Robot on Motor Function Recovery in Patients with Stroke" was retracted in 2023. Reasons: signs of a paper mill; suspected computer-generated content; unreliable results or conclusions; concerns about the data.

### 3.2. Electrophysiological and Imaging Evaluation

After 4 weeks of treatment, the values of the MEP amplitude and latency were significantly improved in both groups (*P* < 0.05), and latency was very significantly improved in the treatment group vs. control (latency, *P* < 0.01; amplitude, *P* < 0.05) (Figure 4(a)). After 4 weeks of treatment, the FA values of the two groups were increased to some extent, but the *P* value of the comparison with baseline was not significant (*P* > 0.05) (Figure 4(b)). Though the FA values in the treatment group were slightly higher, the intergroup comparison was not statistically significant (Figure 4).

## 4. Discussion

### 4.1. Rehabilitation Training with the BCI-LLRR

BCI is a system for communication and control between the human brain and a computer or other electronic system independent of the human peripheral nervous system and muscles. Recently developed human-machine interfaces can be divided into invasive and noninvasive types [5]. The future of research in this area is progressively developing more convenient interfaces, such as those based on the electroencephalogram (EEG), blood oxygen level-dependent functional MRI, steady-state visual evoked potentials, P300 event-related potentials, near-infrared spectroscopy, and others [6–8]. The BCI signals are the normal motor-activity-related changes recorded from the limb movement parts of the brain surface, recognized and translated to corresponding commands for controlling the robot or exoskeleton. This is accomplished through a series of calculations and translations to drive the selected target limb or muscle. Simultaneously, the robot directly stimulates the entire neural network system of the patient by producing sensory and motor feedback [9, 10]. Based on a theory of rehabilitation medicine and the principle of human-machine cooperation, the LLRR provides the patient with an auxiliary training/walking device by simulating the pace of a normal person while standing and utilizes the human body's natural standing antigravity and balance systems [3]. The computer is used to regulate the gait and posture-coordination mechanisms orderly. In the previous research project, we constructed a brain-controlled, active-passive co-stimulation lower limb rehabilitation training robot. Compared with other BCIs, this kind of steady-state motion, combined with mirror-neuron theory and virtual reality technology, can improve the EEG information transmission rate and accuracy stably by means of the limb-feedback training platform and a modified intelligent limb robot system. This system is a much improved realization of a brain-muscle, multisource interaction model [11, 12]. Relying on dynamic feedback to the patient's visual system, the patient's motor imagination, and dynamic compensation of the movement ability of the recuperating limbs, we observed the clinical effects of the BCI-LLRR on patients with stroke. This will provide a theoretical and experimental basis for the study of functional recovery from brain damage.

The article "Effects of a Brain-Computer Interface-Operated Lower Limb Rehabilitation Robot on Motor Function Recovery in Patients with Stroke" was retracted in 2023. Reasons: signs of a paper mill; suspected computer-generated content; unreliable results or conclusions; concerns about the data.

### 4.2. Outcomes

Previous studies have suggested [13, 14] that BCIs and rehabilitation robots can improve the motor function of patients with stroke compared with the groovy rehabilitation therapy (passive activity and targeted physical therapy). In this experiment, the motor function of all patients was improved after 4 weeks of treatment, but the patients who received BCI-LLRR training recovered faster, especially in the Fugl–Meyer lower limb and NIHSS scores. While we found no significant group differences in the upper limb motor function scores, balance and walking function was significantly different between the two groups. This outcome may be related to a recovery law of patients after stroke, which is that the speed of recovery of the legs is usually faster than that of the arms. On the contrary, our results also show that the recovery of leg motor function can be accelerated by the BCI-LLRR. Improvement was also observed in the patients' NIHSS scores because, in noncognitive patients, the scores on limb motor function accounted for 18 points, which places more emphasis on limb muscle strength changes. In addition, we found that training on the BCI-LLRR significantly increased the amplitude of the leg MEP and shortened its latency, which is consistent with the observations of Claflin and Ang [14, 15]. This result is probably due to repeated activation of the fibre-bundle-connected cortical leg movement area. Therefore, the relative improvement in leg motor function observed in the treatment group may be related to an improvement in cortical excitability and an increase in transmission through the descending spinal cord [16, 17].

Previous studies [18, 19] have shown that cortical and spinal cord DTI/DTT images can reflect the integrity of or damage to white matter fibres, and FA data obtained by computer analysis can be used to assess white matter integrity in lesion sites. After 4 weeks of treatment, we found that the FA value of the lesion area was not significantly improved, but cortical motor induction, as indicated by the amplitude and latency of cortical MEPs, had improved significantly. We suggest that, in light of the previous literature, it was logical to evaluate the damage to the CST by investigating the local FA value of stroke lesions, but FA does not completely reflect the functional deficits due to lesions if brain damage is probed externally, as here. This is because injury in the specific parts (such as the primary cortical motor area, the radiation crown area, the internal capsule hind limb zone, and the brain foot area) fails to predict motor deficits consistently. Lindenberg [20] studied the relationship between CST integrity and motor impairment in patients with chronic stroke and found a linear correlation between FA and Fugl–Meyer scores and Wolf scores in the posterior limb zone of the internal capsule. However, Koyama et al. [21] performed a DTI study on patients with haemorrhage in the basal ganglia and found that although the lesions at the inner capsule/radiation crown directly affected the CST, the FA value at the cerebral peduncle level was more accurate in predicting deficits in motor function. In addition, the relationship between the location of the injury and the motor deficit is not exactly the same in patients with haemorrhagic stroke vs. ischemic stroke [22]. Moreover, the integrity of the CST structure represented by the FA value is not equivalent to the completeness of the CST conduction function [23] because the value of the FA is closely related to the integrity of the myelin sheath, fibre compactness, and parallelism, whereas the MEP latency response is merely the fastest time for an action potential to pass through the CST. Of course, a difference in timing between the occurrence of secondary Wallerian degeneration and the timing of abnormality detection in the CST after stroke may also be a factor influencing the consistency of the results.

The article "Effects of a Brain-Computer Interface-Operated Lower Limb Rehabilitation Robot on Motor Function Recovery in Patients with Stroke" was retracted in 2023. Reasons: signs of a paper mill; suspected computer-generated content; unreliable results or conclusions; concerns about the data.

We observed that, after 4 weeks of treatment, the patients' improvement in balancing ability and walking function was not obvious. However, the measures in question may not be directly equivalent to the balance and walking function contributed by the legs, the target of therapy. The therapy is more concerned with the overall ability to move, rather than with the improvement of simple muscle strength, the focus of the measures [24].

### 4.3. Inclusion, Exclusion, and Evaluation Indicators

Currently, researchers have no uniform standard for the inclusion of cases in BCI studies [25]. Studies may be based on different BCI methods (e.g., functional MRI and EEG) and BCI patient requirements are particularly limiting. Some patients are not able to complete treatment, such as those with severe cognitive impairment, those already receiving other BCI-dependent treatments, and those with presence of a neglected side, metal implants in the skull, eye diseases, etc. These may be the future standards of exclusion in this field and can provide a basis for testing in other clinical studies. In addition, there are many types of efficacy evaluation indicators. Generally, these can be divided into three categories [2, 12, 26–28]: clinical scales (subjective evaluation indicators), functional indicators (such as EEG, cortical excitability, and changes in cerebral blood oxygen levels), and structural status indicators (based on DTI/DTT changes in the CST, etc.). These are also the main observation indicators of current brain function research. In our research, these three types of evaluation criteria are combined to ensure that the outcome is very significant. However, it is not clear whether functional indicators can be extended to changes in laboratory-determined serological concentrations of BDNF, VEGF, etc. [29]. These may be among the functional indicators measured in our next clinical trial.

### 4.4. Follow-Up

In the current clinical study on a BCI, it is very important to predict the safety and effectiveness of ongoing therapy through follow-up. However, few patients underwent standard function scale assessments during follow-up, and we found no strong evidence for a benefit of sustained treatment [3, 30]. In our study, we conducted follow-up by telephone and an outpatient protocol with function scale assessments. In the 3 months after discharge, we found that leg motor function, balance ability, walking function, and activities of daily living were significantly better in the treatment group. This result may be related to early recovery of motor function of the leg by use of the rehabilitation robot and provides good evidence for relevance. In the control group, some patients' walking and balance ability had declined at follow-up compared with before discharge, being characterized by difficulty in starting and walking instability. Therefore, use of a BCI-operated LLRR could accelerate the recovery of limb function. The effectiveness of long-term treatment is also noteworthy.

Establishing the safety of clinical applications in the field of BCI-based rehabilitation training is one of the goals of follow-up. Some patients experienced adverse reactions during the trial. For example, temporal visual fatigue and dizziness, which are released rapidly by adjusted the distance between the screen and the patient and to shorten the daily treatment time. However, these patients did not experience similar adverse events during the 3-month follow-up period, indicating that the BCI-operated LLRR is effective for long-term rehabilitation.

The article "Effects of a Brain-Computer Interface-Operated Lower Limb Rehabilitation Robot on Motor Function Recovery in Patients with Stroke" was retracted in 2023. Reasons: signs of a paper mill; suspected computer-generated content; unreliable results or conclusions; concerns about the data.

## 5. Conclusions

Our BCI-operated LLRR can effectively promote the recovery of leg motor function in patients with stroke, which may be related to improving cerebral-cortex excitability and white matter fibre-bundle connectivity. The specific mechanisms of this require further study, such as we could increase the sample size or make a deep exploration in serology.

## Figures and Tables

**Figure 1:** Participant recruitment flow as far as analysis.

**Figure 2:** Changes in motor function scores in participants with stroke before and after treatment with a brain-computer interface-operated lower limb rehabilitation robot. (a) Changes of NHSS before and after treatment. (b) Changes of Fugl–Meyer scores before and after treatment.

**Figure 3:** Changes in the Fugl–Meyer balance scale (Fugl–Meyer BS) and Holden walking function test scores. (a) Changes in the Fugl–Meyer balance scale scores; (b) changes in the Holden walking tests.

**Figure 4:** Changes in the cortical motor evoked potentials (MEPs) and corticospinal tract (CST) structure in the lesion area before and after treatment in both groups. (a) Changes in the cortical motor evoked potentials (MEPs). (b) Trends of the FA value of corticospinal track.

**Table 1:** General data of the two groups ($\bar{x}$ ± *s*).

	Treatment group (*n* = 12)	Control group (*n* = 13)	*P* value
Gender			
Male	7	7	0.8213^*∗*^
Female	5	6	
Age (years)	51.24 ± 7.80	49.56 ± 8.40	0.6101^*∗*^
Duration (weeks)	4.61 ± 1.52	4.85 ± 1.27	0.6714^*∗*^

Hemiplegia side			
Left	5	7	0.5425^*∗*^
Right	7	6	

*Note.* Compared with the control group, ^*∗*^*p* < 0.05.

## Data Availability

The data used to support the findings of this study are available from the corresponding author upon request.
